# The Value of Macrogene Second-Generation Sequencing in the Diagnosis, Guidance of Drug Use, and Efficacy Monitoring of Infectious Pneumonia in Premature Infants

**DOI:** 10.1155/2022/4398614

**Published:** 2022-10-12

**Authors:** LiLi Wang, Ping Zha, YuJuan Wang, Ying Kong, Yu Su, LiYing Dai, Yang Wang

**Affiliations:** Department of Pediatrics, The First Affiliated Hospital of Anhui Medical University, Hefei, Anhui 230000, China

## Abstract

**Objective:**

A group-controlled trial was conducted to explore the value of macrogene second-generation sequencing in the diagnosis, drug use, and efficacy monitoring of infectious pneumonia in premature infants.

**Methods:**

One hundred and thirty-eight premature infants with suspected infectious pneumonia treated in our hospital from March 2019 to June 2022 were selected as subjects. All patients underwent deep phlegm extraction and were randomly divided into two groups. 69 cases of control group were treated with general bacterial and fungal culture. The lavage fluid of the remaining 69 cases of observation group were detected by metagenomic next-generation sequencing (mNGS). The number of diagnosed preterm infants with infectious pneumonia was compared between the two groups, and the diagnostic value of the two methods was analyzed by the receiver operator characteristic (ROC) curve. Then, the differences in clinical efficacy, antimicrobial neonatal intensive care unit (NICU) use time, antimicrobial adjustment frequency, NICU stay time, hospital stay, and serum inflammatory factors were compared between the two groups.

**Results:**

The positive rate of mNGS pathogen detection in the lavage fluid of the observation group was 92.75% (64/69). The positive rate of the culture of the lavage fluid of the control group was 52.17% (36/69). The ROC curve analysis showed that the ROC AUC of traditional culture was 0.752 (95%CI = 0.610-0.894), and that of mNCS was 0.934 (95%CI = 0.854-0.999). In the observation group, there were 35 cases of bacterial infection, 20 cases of fungi, 4 cases of virus, and 5 cases of Chlamydia psittaci. In the control group, 26 cases of bacterial infection and 9 cases of fungi were detected; but viruses and other mycoplasmas could not be detected. After 2 weeks of treatment, the effective rate of the observation group was 95.31%, while that of the control group was 69.44%. The NICU use time, adjustment frequency, NICU stay time, and hospitalization time of antibiotics in the observation group were significantly less than those in the control group, and the difference was statistically significant (*P* < 0.05). After treatment, the levels of serum interleukin-6 (IL-6), procalcitonin (PCT), and hypersensitivity-C-reactive protein (hs-CRP) in observation group were significantly higher than those in control group, and the difference was statistically significant (*P* < 0.05).

**Conclusion:**

mNGS can improve the efficiency of clinical diagnosis of infectious pneumonia in premature infants, effectively improve the detection rate of pathogens and the clinical efficacy of premature infants. At the same time, it can also assist the clinical efficacy monitoring and adjust the treatment plan at any time.

## 1. Introduction

Infectious diseases are currently the diseases with the highest morbidity and mortality in the world. According to epidemiological studies, the most common type of infectious diseases is pulmonary infection (21.8%) [1], which is the main cause of death of infectious diseases. However, pathogenic microorganisms can also be detected by conventional pathogen detection methods, and the two pulmonary imaging findings are also similar, mostly exudative changes. If clinicians cannot correctly differentiate and diagnose infected/noninfectious lung diseases, they will miss the best time for diagnosis and treatment, resulting in the abuse of antibiotics. Therefore, it is very important to guide clinicians to correctly and timely differential diagnosis of pulmonary infection/noninfectious diseases and to formulate a reasonable treatment plan. There are many influencing factors of pulmonary infection in premature infants, which have great complexity and difficulty in clinical prevention and treatment. It has been reported that the younger the gestational age and the lower the body mass of premature infants, the worse the development of premature infants. More tissues and organs are underdeveloped [2].

At present, there are the following detection methods for the diagnosis of pulmonary infectious diseases, including etiology-based detection methods, molecular biology-based detection methods, and immunology-based detection methods [2, 3]. In order to ensure the health and safety of premature infants, nursing or treatment procedures that increase the risk of infection should be avoided [4]. Although these methods have their own obvious advantages, they often expose some weaknesses when dealing with complex infectious diseases, such as tedious detection process, time-consuming, and narrow detection range. As a result, the accuracy of conventional pathogen detection methods is limited [5]. Due to the imperfect development of physiological function and poor immune ability, premature infants have a high risk of pulmonary infection when carrying out protection and treatment measures such as invasive examination and mechanical ventilation. It will have a great adverse impact on the healthy development and life safety of premature infants [6] and cannot be diagnosed and treated in time [7]. Therefore, the application of correct detection methods will help to reduce the misdiagnosis and missed diagnosis rate of clinicians and effectively carry out symptomatic treatment.

Metagenomic next-generation sequencing (mNGS) can directly detect all potential pathogens-bacteria, viruses, fungi, and parasites—in clinical samples without isolation and culture [8]. NGS has the following procedures in detecting pathogens, including sample collection and input: sample types include sputum, nasopharyngeal swabs, airway suction secretions, bronchoalveolar lavage fluid, blood, and tissue. The database should have a complete microbial genome sequence, and the analysis process includes data quality control [9–12]. With the continuous progress of NGS technology, this technology is realizing faster and more comprehensive macrogenomic analysis at lower cost. It is more and more widely used in clinic. However, there are few reports on the application value of macrogene second-generation sequencing technology in the diagnosis, guidance of drug use, and efficacy monitoring of infectious pneumonia in premature infants. This study focused on 138 premature infants with suspected infectious pneumonia treated in our hospital. A group-controlled trial was conducted to explore the value of macrogene second-generation sequencing in the diagnosis, drug use, and efficacy monitoring of infectious pneumonia in premature infants.

## 2. Materials and Methods

### 2.1. General Information

One hundred and thirty-eight premature infants with suspected infectious pneumonia treated in our hospital from March 2019 to June 2022 were selected as subjects. All patients underwent deep phlegm extraction and were randomly divided into two groups. 69 cases of them were treated with general bacterial and fungal culture (control group) and the deep phlegm extraction of the remaining 69 cases were detected by mNGS (observation group). There was no significant difference in the general data between the two groups (*P* > 0.05), as shown in Table 1. All legal guardians of premature infant representatives signed informed consent.

The following are the selection criteria: (1) regardless of sex, all patients who were accompanied by persistent hypothermia or high fever, with apnea or lung moist rales, dyspnea and lung auscultation with wet rales, abnormal leukocyte, and other clinical symptoms; (2) gestational age < 37 weeks; (3) diagnosis gold standard: blood culture and pharyngeal swab smear and culture indicating infection and chest X-ray examination showing patchy infiltration shadow; and (4) complete clinical data.

The following are the exclusion criteria: (1) premature infants with severe heart, liver, renal insufficiency, and malignant tumors; (2) premature infants with pulmonary tuberculosis, congenital bronchial asthma, and other diseases; (3) guardians who refused to have their infants participate; (4) premature infants with other severe infections; (5) premature infants who could not be treated because of drug allergy; and (6) premature infants with serious cardiovascular diseases, arrhythmias, heart failure, and other diseases.

### 2.2. Methods

#### 2.2.1. Diagnostic Method

All patients underwent bronchoalveolar lavage with fiberoptic bronchoscope with more than 5 years of experience. Midazolam was selected for intravenous sedation (instead of midazolam 0.1 mg/kg), endotracheal intubation or nasal endoscopy was performed, and 2% lidocaine was used to topical anesthetize the airway mucosa and segmental bronchi. The top of the bronchoscope was embedded in the branch of the bronchus tree. Inject normal saline at 37°C into the bronchial tree under the following conditions: 1 mL/kg/time, ≤20 mL/time, total volume ≤ 5-10 mL/kg, and suction at 100 mmHg negative pressure. The recovery rate was 40%-60%, and the recovered lavage solution was packed into a sterilized container with a culture sample (sputum 1 mL, bronchoalveolar lavage fluid 5 mL).

For sputum sample detection, at least 2-3 mL sputum was collected and sent to a sterile container for mNGS testing. 600 *μ*L sputum samples and 12 *μ*L sputum IC were collected and mixed in a 2 mL centrifuge tube. After mixing, the wall was broken by biological sample homogenizer (BioPrep-24, Hangzhou Jieyi Technology Co., Ltd., China). After that, 3 min was centrifuged by 12000 rpm centrifuge (LX-200, Haimen Kirin Bell instrument, China), and 400 *μ*L of the supernatant was absorbed into the genomic nucleic acid extraction or purification kit (MD013, Hangzhou Jieyi Biotechnology Co., Ltd., China). After that, reagents were added to the cartridge and finally put into the nucleic acid automatic detection reaction system construction system (NGSmaster™ library preparation, MAR002, Hangzhou Jieyi Biotechnology Co., Ltd.). In the abovementioned construction system, the DNA library is established after automatic nucleic acid extraction, endonuclease digestion, end repair, end adenylation, node ligation, and other procedures. The established library was quantitatively analyzed and summarized by real-time PCR (KAPA). The quantitative DNA library is sequenced in the illumina Nextseq system (Inman Inc., USA) with high throughput. The original data obtained by sequencing first filtered the low-quality sequences, then filtered the human-derived sequences (GRCh38.p13), and compared the remaining sequences with the reference microbial Gene Database (NCBINt, GenBank, and in-house curated genomic database) to determine the microbial species and sequence count.

For the detection of bronchoalveolar lavage fluid samples, respiratory physicians lavaged the focus under bronchoscope according to the lung imaging findings of the patients and obtained at least 2-3 mL bronchoalveolar lavage fluid (BALF) into aseptic containers for mNGS testing. Samples of lavage fluid and brush were sent to the laboratory for microbiological detection at the same time. In addition, the bacterial and fungal smears and culture of sputum were routinely detected in patients with pulmonary infection. 1.2 mL bronchoalveolar lavage fluid samples and 12 *μ*L bronchoalveolar lavage fluid IC were mixed in a 2 mL centrifuge tube, and then, the wall was broken by a biological sample homogenizer (BioPrep-24, Hangzhou Ausheng, China). After that, 12000 rpm was centrifuged for 3 min (LX-200, Haimen Qilin Bell instrument, China); absorb 400 *μ*L of the supernatant to the genomic nucleic acid extraction or purification kit (MD013, Hangzhou Jieyi Biotechnology Co., Ltd., China), and add other corresponding reagents to the card box as required, and finally put it into the automatic nucleic acid detection reaction system construction system (NGSmaster™ library preparation, MAR002, Hangzhou Jieyi Biotechnology Co., Ltd., China). In the above-mentioned construction system, the DNA library is established after automatic nucleic acid extraction, endonuclease digestion, end repair, end adenylation, node ligation, and other procedures. The established library was quantitatively analyzed and summarized by real-time PCR (KAPA). The quantitative DNA library is sequenced in the illumina Nextseq system (Inman Inc., USA) with high throughput. The original data obtained by sequencing first filtered the low-quality sequences, then filtered the human-derived sequences (GRCh38.p13), and compared the remaining sequences with the reference microbial Gene Database (NCBINt, GenBank, and in-house curated genomic database) to determine the microbial species and sequence count.

#### 2.2.2. Treatment Scheme

The patients in the control group were treated with routine treatment, including warmth, oxygen inhalation, sputum suction, and anti-infection. Cefotaxime sodium was mainly selected for anti-infection. The dose of cefotaxime sodium was 50 mg/kg each time, and the dose of cefotaxime sodium could be increased to 200 mg/(kg·d) by intravenous drip 3 times a day for patients with severe infection. The curative effect was evaluated after continuous treatment for 2-3 weeks. The medication regimen could be adjusted continuously according to the patient's condition.

On the basis of the control group, the patients in the observation group adjusted the anti-infective regimen according to the mNGS results of bronchoalveolar lavage fluid. Patients with pneumonia caused by bacteria can be treated with antibiotics, such as cefaclor, amoxicillin, azithromycin, meropenem, and cefuroxime. Patients with pneumonia caused by virus can be treated with detoxification and antiviral drugs. Patients with pneumonia caused by mycoplasma and chlamydia can be treated with erythromycin, meropenem, and azithromycin. The specific medication plan of the patients in the observation group should be adjusted according to the severity of the patient's condition, body weight, drug allergy, and other indexes. The curative effect was evaluated after continuous treatment for 2-3 weeks. The medication plan could be adjusted continuously according to the changes of the patient's condition during the treatment period.

### 2.3. Observation Index

#### 2.3.1. Physical Examination of Pathogen

The detection rate and distribution of pathogens were compared between the two groups. Pathogen physical examination rate = (number of pathogen positive cases/total number of cases in this group) × 100%.

#### 2.3.2. Clinical Curative Effect

The third-grade standard was used to evaluate the clinical curative effect. Two weeks after treatment, according to the standard published by Jing [13], it was divided into three levels, consisting of markedly effective, effective, and ineffective, and the total effective was the total effective. Effective rate = (number of significantly effective cases + number of effective cases)/total number of cases × 100%. The 28-day mortality of the patients was calculated.

#### 2.3.3. The Antimicrobial NICU Use Time, Adjustment Frequency, NICU Stay Time, and Hospital Stay between the Two Groups

At the end of treatment, the neonatal intensive care unit (NICU) use time, adjustment frequency, NICU stay time, and hospitalization time of the two groups were compared.

#### 2.3.4. Cytokine Level

IMMULITE/IMMULIE1000 analyzer, immune scattering turbidimetry, sandwich, and chemiluminescence methods were used to detect serum cytokines (hs-CRP, PCT, and IL-6). The detection process was strictly in accordance with the instructions, before treatment and 2 weeks after treatment. All the kits were purchased from SIEMENS company in Germany. According to the operation flow of the manufacturer's instructions, the processed samples were sent to the analyzer for detection. The corresponding cytokine concentration was recorded.

### 2.4. Statistical Analysis

The data were analyzed by SPSS23.0 software. The normal distribution of measurement data was expressed by the mean ± standard deviation, a *t*-test was used for the comparison between groups, a frequency method was used for counting data, a *χ*^2^ test was used for comparison between groups, and a bilateral test was used for all statistical tests. The ROC curve of the measurement index is drawn, the AUC value is calculated, and the prediction performance of each parameter is analyzed and evaluated. According to statistics, the actual range of AUC value is 0.5-1. The diagnostic value of AUC was lower when 0.5~0.7, moderate when AUC was 0.7~0.9, and higher when AUC > 0.9. The Youden index was used to determine the best predictive standard value of each parameter and its accuracy, sensitivity, specificity, PPV, NPV, and *P* < 0.05. There were significant differences in statistics.

## 3. Results

### 3.1. Analysis of Clinical Data of Two Groups of Premature Infants

First, we analyzed the clinical data of 138 premature infants. The comparison of clinical data between the two groups is shown in Table 1. There was no significant difference in clinical data between the two groups (*P* > 0.05).

### 3.2. Diagnostic Value of Traditional Culture and mGCS Detection in Preterm Infants with Infectious Pneumonia

The positive rate of mNGS pathogens in lavage fluid was 92.75% (64/69) in the observation group and 52.17% (36/69) in the control group. We further analyzed the diagnostic value of traditional culture and mNCS detection in preterm infants with infectious pneumonia by ROC curve. The results showed that the ROC AUC of traditional culture was 0.752 (95%CI = 0.610~0.894) and the ROC AUC of mNCS was 0.934 (95%CI = 0.854~0.999). All results are shown in Figure 1.

### 3.3. Application Effect of Traditional Culture and mGCS Detection in Pathogen Detection of Infectious Pneumonia in Premature Infants

The application effect of traditional culture and mGCS detection in pathogen detection of infectious pneumonia in premature infants was analyzed. 35 cases of bacteria were detected in the observation group, of which Klebsiella pneumoniae (15.63%) and Acinetobacter baumannii (12.50%) were the highest. There were 20 cases of fungi, of which the detection rate of Pneumocystis carinii was the highest (12.50%). The detection rate of Candida albicans and Aspergillus fumigatus was 7.81%. There were 4 cases of virus, of which human sporovirus 5 was the main type of virus with a detection rate of 3.13%. There were 5 cases of Chlamydia psittaci, 1 case of Mycobacterium tuberculosis, and 1 case of Mycobacterium Kansas. A total of 26 cases of bacteria were detected in the control group, of which Acinetobacter baumannii was the highest, followed by Klebsiella pneumoniae, Pseudomonas aeruginosa, Staphylococcus aureus, Streptococcus pneumoniae, and Serratia marcescens. Nine cases of fungi, Candida albicans (13.89%), and Aspergillus fumigatus (11.11%) failed to detect virus and other mycoplasma. All results are shown in Table 2.

### 3.4. Comparison of Clinical Efficacy between the Two Groups

The clinical effects of the two groups were compared. After 2 weeks of treatment, 27 cases were significantly effective, 30 cases were effective, and 3 cases were ineffective in the observation group. The effective rate was 95.31%. The control group was significantly effective in 10 cases, effective in 15 cases, and ineffective in 11 cases. The treatment effective rate was 69.44%, and the difference was statistically significant (*P* < 0.05). All results are shown in Figure 2.

### 3.5. The Antimicrobial NICU Use Time, Adjustment Frequency, NICU Stay Time, and Hospital Stay between the Two Groups

Comparing the NICU use time, adjusted frequency, NICU stay time, and hospitalization time of the two groups of patients, the observation group was significantly shorter than the control group in terms of antibiotic NICU use time, adjusted frequency, NICU stay time, and hospital stay, and the difference was statistically significant (*P* < 0.05). All results are shown in Table 3.

### 3.6. Comparison of Cytokine Levels between the Two Groups after Treatment

After treatment, the serum levels of IL-6, PCT and hs-CRP in both groups decreased significantly, and the difference was statistically significant (*P* < 0.05). The observation group was significantly lower than the control group, and the difference was statistically significant (*P* < 0.05). All the results are shown in Table 4.

## 4. Discussion

As the normal physiological mechanism of premature infants cannot play an effective role, the sensitivity to the external environment is high. It is difficult to adjust and adapt, and the immune ability to bacteria is poor [14]. Respiratory function is in the tubule stage with low secretion of active substances on the lung surface, poor pulmonary compliance, and imperfect independent breathing [15, 16]. The need for the establishment of artificial channels and mechanical ventilation and other invasive means greatly increases the risk of respiratory infection in premature infants but also have the risk of inhibiting lung development, leading to chronic respiratory sequelae [17, 18].

Early identification of infectious pathogens and targeted anti-infection is the key to the treatment of infectious pneumonia. Traditional pathogen culture requires high conditions, long cycle, and low positive rate, and the use of antibiotics affects its culture. A large number of clinical data show that the inability to identify the infectious pathogen of infectious pneumonia as soon as possible is one of the important reasons for the high mortality of this kind of disease [19]. The unknown pathogen of infection has seriously affected the effect of empirical anti-infective treatment [20]. Therefore, there is an urgent need for new detection techniques to quickly and accurately find infectious pathogens and give accurate anti-infective treatment.

In this study, the detection rate of mNGS pathogens in lavage fluid of the observation group was 92.75%, which was significantly higher than that of the control group (52.17%). This study systematically compared mNGS and traditional culture methods and found that mNGS has advantages in many aspects. First, mGCS has higher diagnostic value for infectious pneumonia in premature infants. The ROC curve analysis showed that the traditional culture ROCAUC was 0.752, which was significantly lower ROCAUC0.934 which was detected in mNCS. In addition, mNGS has a clear advantage in detecting pathogens such as Klebsiella, anaerobes, Pseudomonas, viruses, and mycoplasma. The results of this study showed that the proportion of pathogens in the observation group was bacteria, fungi, viruses, and other pathogens from high to low. And most of the bacteria were gram-negative bacteria. Pseudomonas aeruginosa, Acinetobacter baumannii, and Klebsiella pneumoniae were the main gram-negative bacteria. Staphylococcus aureus was the main gram-positive bacteria. Therefore, anti-Pseudomonas aeruginosa *β*-lactam drugs should be considered in the empirical anti-infection of infectious pneumonia in premature infants and vancomycin should be added if necessary. 20 cases of fungi were detected in the observation group. We found that most of these premature infants had a history of hormone treatment, so we should routinely improve G test and GM test and experience antifungal therapy as soon as possible. In addition, the observation group also detected rare pathogens such as Nucasmella, Mycobacterium tuberculosis, and Mycobacterium Kansas. MNGS can sequence hundreds of thousands to millions of DNA molecules at one time and can detect the gene sequences of culturable and unculturable microorganisms, bypassing the process of microbial isolation and culture. It has the characteristics of high positive rate, high speed, and high sensitivity in pathogen detection [21–23]. The traditional culture conditions of these pathogens are very high, which generally need to be cultivated in tuberculosis hospitals, suggesting that mNGS can improve the detection rate of rare pathogens.

In this study, 5 premature infants with severe pneumonia were finally diagnosed with Chlamydia psittaci infection by mNGS. It is reported that Chlamydia psittaci pneumonia accounts for about 1% of community-acquired pneumonia [24]. The sensitivity and specificity of traditional serological test or PCR test are not high, and the pathogen is extremely difficult to culture. In the past, most patients were missed or misdiagnosed due to the limitation of detection conditions. With the popularization of mNGS technology, the disease is reported more and more [25, 26]. The virus is extremely difficult to cultivate in the ordinary laboratory of the hospital, and the diagnosis of viral pneumonia has always been a clinical problem. Clinical diagnosis combined with medical history and chest CT manifestations for empirical diagnosis, the accurate diagnosis, and treatment of patients are seriously lagging behind [27–30]. In this study, no virus was detected in the control group, indicating that mNGS has a good effect in the diagnosis of virus infection.

Most of the pathogenic bacteria in patients with pneumonia are unknown. Patients with severe pneumonia often require long-term, high-dose broad-spectrum antibiotics. This phenomenon has led to the rising rate of antibiotic resistance of pathogenic bacteria, which is an urgent problem to be solved globally. Our findings showed that early identification of pathogens and timely adjustment of treatment plan through mNGS could reduce the adjustment frequency and NICU use time of antibiotics, which will provide a new direction for the management of antibiotics. With the progress of technology, we expect that mNGS can detect drug resistance genes and better guide clinical anti-infective treatment. At the same time, it was found that the effective rate of clinical treatment in the experimental group was higher. The length of stay and the cost of hospitalization were lower, which improved the prognosis of patients and reduced their economic burden. The above data analysis suggested that mNGS played a positive role in guiding the choice of treatment for premature infants with infectious pneumonia. The limitation of the mNGS method for the diagnosis of infectious pneumonia is that this technology is affected by the equipment of the hospital, because some hospitals do not routinely use the mNGS method in the diagnosis of infectious pneumonia. This study still has some shortcomings. Firstly, the quality of this study is limited due to the small sample size we included in the study. Secondly, this research is a single-center study, and our findings are subject to some degree of bias. Therefore, our results may differ from those of large-scale multicenter studies from other academic institutes. This research is still clinically significant, and further in-depth investigations will be carried out in the future.

To sum up, mNGS is of high value in the diagnosis of infectious pneumonia in premature infants. It can significantly improve the detection rate of pathogens in severe pneumonia and can adjust the treatment plan according to the pathogen detection results of mNGS. It can shorten the time of use of antibiotics and adjust frequency and hospital stay.

## Figures and Tables

**Figure 1:** ROC curve of traditional culture and mGCS detection in the diagnosis of infectious pneumonia in premature infants.

**Figure 2:** Comparison of clinical efficacy between the two groups.

**Table 1:** The clinical data of 138 premature infants [*n*/%].

Basic data	Research group (*n* = 69)	Control group (*n* = 69)	*χ* ^2^/*t*	*P*
Gender			0.727	0.394
Male	30 (43.48)	35 (50.72)		
Female	39 (56.52)	34 (49.28)		
Gestational age (weeks)	30.81 ± 3.16	30.93 ± 3.26	0.220	0.827
Body weight (kg)	1.91 ± 0.68	1.85 ± 0.62	0.542	0.589
Mode of production			0.267	0.606
Cesarean section	41 (59.42)	38 (55.07)		
Natural delivery	28 (40.58)	31 (44.93)		
Premature rupture of membranes			1.451	0.228
Yes	43 (62.32)	36 (52.17)		
No	26 (37.68)	33 (47.83)		
1 min Apgar scoring			0.116	0.733
≤7 points	35 (50.72)	37 (53.62)		
>7 points	34 (49.28)	32 (46.38)		
Coma			0.038	0.845
Yes	17 (24.64)	18 (26.09)		
No	52 (75.36)	51 (73.91)		

**Table 2:** Analysis and comparison of pathogen physical examination between the two groups (*n*/%).

Pathogen	Observation group (*n* = 64)	Control group (*n* = 36)
Bacteria		
Pseudomonas aeruginosa	5 (7.81)	5 (13.89)
Klebsiella pneumoniae	10 (15.63)	6 (16.67)
Acinetobacter baumannii	8 (12.50)	8 (22.22)
Streptococcus pneumoniae	2 (3.13)	2 (5.56)
Staphylococcus aureus	5 (7.81)	5 (13.89)
Legionella pneumophila	2 (3.13)	—
Nocardia	1 (1.56)	—
Serratia marcescens	1 (1.56)	1 (2.78)
Burkholderia cepacia	1 (1.56)	—
Fungus		
Candida albicans	5 (7.81)	5 (13.89)
Pneumocystis Yersini	8 (12.50)	—
Aspergillus fumigatus	5 (7.81)	4 (11.11)
Virus		
Human spore virus type 1	1 (1.56)	—
Human sporrash virus 5	2 (3.13)	—
Cytomegalovirus	1 (1.56)	—
Chlamydia psittaci	5 (7.81)	—
Mycobacterium tuberculosis	1 (1.56)	—
Mycobacterium Kansas	1 (1.56)	—

**Table 3:** The antimicrobial NICU use time, adjustment frequency, NICU stay time, and hospital stay between the two groups [$\bar{x}\pm s$].

Grouping	*N*	Antimicrobial NICU use time (d)	Adjustment frequency of antibiotics (times)	NICU residence time (d)	Hospitalization time (d)
Observation group	64	16.47 ± 2.68	2.41 ± 0.51	10.65 ± 4.46	18.58 ± 2.66
Control group	36	19.43 ± 3.62	3.77 ± 0.62	14.78 ± 5.51	21.96 ± 4.43
*t*		4.659	11.830	4.078	4.772
*P*		<0.05	<0.05	<0.05	<0.05

**Table 4:** Cytokine levels between the two groups after treatment [$\bar{x}\pm s$].

Grouping	*N*	IL-6 (ng/mL)		PCT (ng/mL)		hs-CRP (mg/L)	
		Before treatment	After treatment	Before treatment	After treatment	Before treatment	After Treatment
Observation group	64	95.22 ± 15.06	73.76 ± 7.01^∗^	25.27 ± 1.93	12.62 ± 1.88^∗^	29.96 ± 6.66	18.42 ± 4.12^∗^
Control group	36	95.39 ± 15.33	80.97 ± 14.32^∗^	25.36 ± 2.01	20.24 ± 0.84^∗^	30.10 ± 6.74	25.18 ± 6.74^∗^
*t*		0.054	3.380	0.221	27.922	0.100	6229
*P*		>0.05	<0.05	>0.05	<0.05	0.920	<0.05

^∗^Compared with that before treatment, the difference was statistically significant (*P* < 0.05).

## Data Availability

The datasets used and analyzed during the current study are available from the corresponding author upon reasonable request.
